# Efficacy and Safety Differences between Domestic Paclitaxel Drug-Coated Balloons and Metal Bare Stents in the Treatment of ASO of Femoral-Popliteal Arteries Type IIA–C

**DOI:** 10.1155/2022/6817838

**Published:** 2022-07-06

**Authors:** Fuqing Wei, Fenglei Huang, Fengkui Cui

**Affiliations:** ^1^Department of Vascular Surgery, Daqing Oilfield General Hospital, Daqing, China; ^2^Interventional Operating Room, Daqing Oilfield General Hospital, Daqing, China

## Abstract

The aim in this study was to investigate the efficacy and safety of domestic paclitaxel-coated balloon (DCB) and bare metal stent (BMS) in the treatment of Transatlantic Cooperative Organization Consensus II (ASC II) types A–C femoral-popliteal arteriosclerosis obliterans (ASO). A total of 103 patients with ASC II A–C femoropopliteal ASO, who received treatment in our hospital from March 2020 to March 2021, were retrospectively selected and divided into the DCB group (*n* = 56) and BMS group (*n* = 47), according to treatment methods. The general clinical data and surgical results were compared between the two groups. The patients were followed up, and the primary patency rate, restenosis rate, freedom from target lesion revascularization (f-TLR), and limb preservation rate were recorded. The liver and kidney functions before and after operation and the occurrence of major postoperative adverse events were recorded. The operation was successful in both groups. The minimum diameter of the DCB group was smaller than that of the BMS group after treatment (*P* < 0.05). At 6 and 12 months after operation, the Rutherford classification decreased and ABI index increased in both groups (*P* < 0.05), but there was no significant difference (*P* > 0.05). At 6 and 12 months after surgery, f-TLR was significantly higher in the DCB group than in the BMS group (*P* < 0.05); at 12 months after surgery, the restenosis rate was lower in the DCB group than in the BMS group (*P* < 0.05). There was no significant difference in the primary patency rate and limb preservation rate at 6 and 12 months after operation between the two groups (*P* > 0.05). Before and after operation, there was no significant difference in liver and kidney function between the two groups (*P* > 0.05). Within 12 months after surgery, 1 patient in the DCB group developed puncture site hematoma 3 days after surgery, and 1 patient in the BMS group developed acute thrombosis 1 day after surgery, and no intervention-related deaths occurred. Domestic paclitaxel DCB can achieve better f-TLR and lower restenosis rate than BMS in the treatment of type II A–C femoral-popliteal artery ASO. Short-term and medium-term efficacy and safety are comparable to BMS.

## 1. Introduction

Arteriosclerosis obliterans (ASO) is a chronic progressive disease of the lower extremities due to arterial stenosis or occlusion, which is clinically characterized by intermittent claudication, pain, and ulcers in the lower extremities, and in severe cases, amputation or even death [1, 2]. The femoral-popliteal artery is a common site of ASO, and for patients with Transatlantic Collaborative Group Consensus II (ASC II) classification A–C, the guidelines recommend percutaneous transluminal angioplasty (PTA) as the treatment of choice, but the restenosis rate after PTA is high and the clinical effect is limited [3, 4]. Bare metal stents (BMS) as a remedy after PTA can significantly improve the clinical outcome of PTA alone, but the stimulation of the intima during the application of BMS can lead to intimal elastosis, affecting the medium to long-term patency of the artery and even causing the patient to suffer from lower limb ischaemia again due to stent fracture [5, 6]. In order to ensure the long-term effectiveness of endovascular treatment and reduce the incidence of postoperative restenosis, drug-coated balloon (DCB) has been gradually applied in clinical practice. Foreign studies [7] have shown that the primary patency rate of DCB in the treatment of femoral-popliteal ASO is 83.2%, which can obtain satisfactory clinical efficacy. However, in China, whether domestic DCB also has better clinical efficacy and safety, it needs to be further explored. In this study, we compared the efficacy and safety of domestic paclitaxel DCB and BMS in the treatment of ASC IIA–C femoral-popliteal ASOs in order to provide a reference for the selection of treatment options for this type of patients in clinical practice.

## 2. Patients and Methods

### 2.1. Patients

This study was approved by the Ethics Committee of Daqing Oilfield General Hospital. Informed consents were obtained from all participants before the study. 103 patients with ASC II A–C femoral-popliteal artery ASO who received treatment in our hospital from March 2020 to March 2021 were retrospectively selected. The inclusion criteria was as follows: all patients' clinical examination was in accordance with the diagnostic criteria of ASO [8] and confirmed by CT arteriography (CTA) or magnetic resonance angiography (MRA); the diseased vessels were superficial femoral artery and/or above-the-knee popliteal artery; ASC II classification was A–C; Rutherford classification was 2–5; the diameter of the reference vessel was 4–7 mm; and expected survival time was ≥12 months. The exclusion criteria were as follows: history of stroke or ST-segment elevation myocardial infarction within 3 months before enrollment; patients allergic to paclitaxel drugs; patients with anticoagulant or antiplatelet contraindications; and patients who fail to open the target lesion area during surgery. The patients were divided into the DCB group (*n* = 56) and BMS group (*n* = 47) according to different treatment modalities.

### 2.2. Treatment Method

Preoperative preparation: after admission, all patients perfected routine examinations, like blood routine, electrocardiogram (ECG), cardiac ultrasound, and X-ray to evaluate surgical risks, and were told to strictly quit smoking. 3 days before operation, the patients were given “dual antiplatelet” (aspirin 100 mg/d, clopidogrel tablets 75 mg/d) and rosuvastatin calcium tablets (20 mg/d) for treatment and hypoglycemic, antihypertensive, anti-infective, and other symptomatic treatments for complications.

Surgical treatment: the patient was placed in the supine position, the ipsilateral or contralateral femoral artery and brachial artery approach were selected, the puncture site was routinely disinfected and draped, and the puncture site was planned for local anesthesia with 2% lidocaine; after successful puncture by the Seidinger method, a 5F or 6F arterial sheath was placed and systemic heparinization was performed (70 IU/kg, intraoperative heparin supplementation could be performed if necessary, and the supplementary dose was 50% of the first dose). Angiography was performed using an angiographic machine (Siemens Artis DTA, Siemens, Germany) to identify the location, extent, length, and outflow tract of the lesion, with angiographic parameters 71.4 kV, 51880 mAs and fluoroscopic parameters 73.5 kV, 1273.5 mAs. The balloon model was determined according to the angiographic performance. The common balloon was selected first for predilatation, with the dilatation time of 2-3 min; if multiple balloons were required for continuous dilatation, it should be noted that there shall be 10 mm overlap between two balloons. After the completion of predilatation, the DCB group received dilatation with domestic paclitaxel DCB (Beijing Xerida Medical Technology Co., Ltd., Beijing, China). The balloon used 3 mg/mm^2^ paclitaxel coating as the antiproliferative agent, magnesium stearate as the carrier matrix, the diameter was 4-5 mm, and the expansion time was 3–5 min. To avoid the loss of the target area, the DCB selected 10 mm more proximal and distal to the lesion. The BMS group received vascular recanalization treatment with bare metal stents. The specific type and model of the stent were determined by the operator. In order to avoid the loss of the target area, the stent length should exceed 10 mm proximal and distal to the lesion, respectively; if multiple stents are needed to be placed, the stent should be placed in the order of first distant from the puncture site and then close to the puncture site. Angiography was performed again after the completion of dilatation. If poor stent expansion (<50%), flow-limiting dissection, or residual stenosis >50% occurred during the operation, a rescue stent was placed until the contrast medium was well developed, without vascular recoil or arterial segment thrombosis formed in the distal outflow tract. At the end of the operation, the catheter was removed, and local compression hemostasis was performed for 30 minutes, and compression bandaging was performed at the puncture site.

Postoperative treatment: postoperative limb on the punctured side was braked for 12 h or more, postoperative low molecular heparin sodium (4000 U) was routinely given subcutaneously 2 times/d for 7 d; oral poliovirus (75 mg) was given once/d for 3 months; long-term aspirin was given once/d (100 mg).

The patients returned to the hospital for reexamination at 1 month, 3 months, 6 months, and 12 months after operation for clinical evaluation, arterial CTA, and Doppler ultrasonography.

### 2.3. Observation Indicators

(1) General clinical data: general clinical data such as gender, age, underlying diseases, smoking history, history of cerebral infarction, course of disease, ASC II classification, lesion length, and stenosis rate were collected. (2) Surgical effect: the success rate of operation, Rutherford classification, and ankle-brachial index (ABI) before operation and 6 months and 12 months after operation were recorded. (3) Follow-up results: the primary patency rate, freedom from target lesion revascularization (f-TLR), restenosis rate, and limb preservation rate were recorded at 6 and 12 months after operation. Restenosis was defined as the degree of stenosis of the target lesion >50% of the reference diameter or the target lesion peak blood flow ratio >2.4; the rate of avoiding amputation above the ankle level was considered as the rate of limb preservation. (4) Liver and kidney function: serum samples were taken from patients before surgery and 6 months after surgery, and alanine aminotransferase (ALT), aspartate aminotransferase (AST), serum creatinine (Scr), and blood urea nitrogen (BUN) levels were measured using an automatic biochemical analyzer (Modular P800, Roche, Switzerland). (5) Occurrence of major adverse events: the major adverse effects include postoperative puncture site complications, intraoperative distal embolism, early thrombosis, and intervention-related death.

### 2.4. Statistical Analysis

In this study, Statistical Product and Service Solutions (SPSS) 25.0 software (IBM, Armonk, NY, USA) was used as a statistical analysis tool, the enumeration data were described in the form of (*n*)%, the *χ*^2^ test or Fisher's exact probability test was performed, the rank sum test was used for grade data, and measurement data were analyzed by (*x̅* ± *s*), which were expressed and the *t*-test was used, and *P* < 0.05 was considered statistically significant.

## 3. Results

### 3.1. General Clinical Data in the Two Groups

The general clinical data of the two groups were not significantly different (*P* > 0.05), with comparability (Table 1).

### 3.2. Surgical Results in the Two Groups

The operation was successful in both groups. There was 1 case of flow-limiting dissection in the DCB group, and rescue stent was placed during the operation. The minimum diameter after treatment in the DCB group was smaller than that in the BMS group, and the difference had a statistical significance (*P* < 0.05). There was no significant difference in Rutherford classification and ABI index between the two groups before operation (*P* > 0.05). At 6 and 12 months after operation, Rutherford classification decreased and ABI index increased in the two groups (*P* < 0.05), but there was no significant difference (*P* > 0.05) (Table 2).

### 3.3. Follow-Up Results in the Two Groups

At 6 and 12 months after surgery, f-TLR was significantly higher in the DCB group than in the BMS group (*P* < 0.05); at 12 months after surgery, the restenosis rate was lower in the DCB group than in the BMS group (*P* < 0.05). There was no significant difference in the primary patency rate and limb preservation rate at 6 and 12 months after operation between the two groups (*P* > 0.05) (Table 3).

### 3.4. Liver and Kidney Functions before and after Surgery in the Two Groups

Before and after surgery, ALT, AST, Scr, and BUN levels did not change significantly in both groups (*P* > 0.05) (Table 4).

### 3.5. The Incidence of Major Adverse Events in the Two Groups

Within 12 months after operation, 1 patient in the DCB group had puncture site hematoma 3 days after operation, which was improved after conservative treatment; 2 patients had increased skin temperature 15 days and 1 month after operation, which was gradually subsided; no thrombosis, intervention-related death, and other serious adverse events occurred. One patient in the BMS group developed acute thrombosis 1 day after surgery, and recanalization was achieved after aspiration of mechanical thrombus removal; no intervention-related death occurred.

## 4. Discussion

With the improvement of living standards and the aggravation of the aging population, the incidence of ASO is increasing year by year and has become one of the major diseases threatening the life safety of patients. As a classic intramural treatment, BMS materials have the advantages of flexibility, high biocompatibility, and good support and have good clinical efficacy in improving the short-term patency rate after PTA and improving the patient's postoperative motor function [9]. With the development of endovascular treatment technology, the advantages of DCB in the clinical treatment of ASO are highlighted. DCB technology applies antivascular intimal hyperplasia drugs to the balloon surface, which can reduce restenosis by inhibiting the proliferation of smooth muscle and fibroblasts [10]. A large foreign randomized controlled trial [11] confirmed that patients treated with DCB can achieve higher long-term patency rates and can significantly reduce the placement of stents compared with PTA. Paclitaxel is a commonly used antiproliferative drug in clinical practice, which has the advantages of solubility, good antiproliferative effect, and continuous effect. However, there is no sufficient clinical evidence-based data on the efficacy and safety of domestic paclitaxel DCB compared with BMS.

This study compared the efficacy and safety of domestic paclitaxel DCB and BMS in the treatment of ASC IIA–C femoropopliteal ASO. At 6 and 12 months after operation, there was no significant difference between the two groups, suggesting that domestic paclitaxel DCB is equivalent to BMS in improving Rutherford classification and ABI index. A previous study [12] analyzed the efficacy of DCB in the treatment of elderly patients with long-segment ASO lesions and found that the short-term and midterm efficacies of DCB in the treatment of long-segment ASO lesions were not inferior to that of BMS. It was considered that DCB could rapidly release the coating drug to the intima of the diseased vessel through balloon dilatation, which not only reduced the stimulation of foreign body implantation to the wall but also avoided the risk of restenosis after BMS. This study also found that the minimum diameter after treatment in the DCB group was smaller than that in the BMS group, which was considered to be related to the reballoon dilatation without stent deployment after stent release in the BMS group. In addition, 1 patient in the DCB group in this study still underwent bailout stent implantation due to flow-limiting dissection, which was considered to be related to the patient's lesion time and increased need for bailout stents, and may also be related to the operator's early assessment of the degree of calcification, the severity of plaque tear, and elastic recoil [13]. Therefore, before clinical DCB treatment, the patient's condition should be fully assessed and the indications for DCB should be strictly grasped.

The coating drug paclitaxel is highly lipophilic and can be rapidly absorbed by the tissue of vascular wall, reducing the drug loss caused by blood flow scouring and maintaining a high drug concentration in a short time, thus continuously exerting the effect of inhibiting intimal hyperplasia [14]. In addition, the rapid release and absorption of paclitaxel can inhibit the delay of vascular endothelialization and reduce re-revascularization [15]. In terms of safety, the liver and kidney functions of the two groups were comparable. There was 1 patient with puncture site hematoma in the DCB group and 1 patient with acute thrombosis in the BMS group, no intervention-related death occurred, and the patients with adverse events were improved after symptomatic treatment, suggesting that the safety of domestic paclitaxel DCB is equivalent to that of BMS. This study is a single-central randomized controlled study with a small sample size, and the results obtained need to be further confirmed in a large multicentral, randomized, and double-blind controlled study.

## 5. Conclusion

In summary, domestic paclitaxel DCB can achieve better f-TLR and lower restenosis rate than BMS in the treatment of type IIA–C femoral-popliteal ASOs, with no significant difference in short and midterm efficacies and safety compared with BMS.

## Figures and Tables

**Table 1:** Comparison of general clinical data between the two groups (*n* (%), $\bar{x}\pm s$).

Metrics		DCB group (*n* = 56)	BMS group (*n* = 47)	*t*/*χ*^2^	*P*
Sex	Male	41 (73.21)	38 (80.85)	0.834	0.361
	Female	15 (26.79)	9 (19.15)		

Age (years)		68.75 ± 9.24	67.28 ± 10.23	0.766	0.446

Underlying disease	Diabetes	34 (60.71)	26 (55.32)	0.306	0.580
	Hypertension	36 (64.29)	32 (68.09)	0.164	0.685
	Hyperlipidemia	29 (51.79)	26 (55.32)	0.128	0.720

Smoking history		25 (44.64)	23 (48.94)	0.273	0.602

History of cerebral infarction		8 (14.29)	5 (10.64)	0.308	0.579

Disease duration (years)		1.31 ± 0.24	1.28 ± 0.43	0.446	0.657

ASC II classification	A	15 (26.79)	11 (23.40)	0.183	0.913
	B	19 (33.93)	16 (34.04)		
	C	22 (39.29)	20 (42.56)		

Lesion length (mm)		146.78 ± 79.45	163.24 ± 65.39	1.134	0.260

% stenosis		94.73 ± 4.21	93.68 ± 4.19	1.2163	0.209

**Table 2:** Comparison of surgical results between the two groups (*n* (%), $\bar{x}\pm s$).

Metrics		DCB group (*n* = 56)	BMS group (*n* = 47)	t/*χ*^2^	*P*
Procedure success		56 (100.00)	47 (100.00)		

Place bailout stent		1 (1.79)	0 (0.00)	—	1.000^*∗*^

Minimum diameter after treatment (mm)		3.68 ± 0.53	4.49 ± 0.61	7.211	<0.001

Rutherford classification	Preoperation	4.09 ± 0.53	4.02 ± 0.52	0.673	0.502
	6 months after operation	1.73 ± 0.48^#^	1.76 ± 0.57^#^	0.290	0.772
	12 months after operation	1.45 ± 0.75^#^	1.51 ± 0.66^#^	0.427	0.670

ABI	Preoperation	0.43 ± 0.09	0.41 ± 0.08	1.181	0.240
	6 months after operation	0.86 ± 0.09^#^	0.83 ± 0.11^#^	1.522	0.131
	12 months after operation	0.89 ± 0.12^#^	0.86 ± 0.09^#^	1.412	0.161

^*∗*^Fisher's exact probability test; compared with the same group, P < 0.05; ^#^ indicates P < 0.05, compared with the preoperation group.

**Table 3:** Comparison of follow-up results between the two groups (*n* (%)).

Metrics		DCB group (*n* = 56)	BMS group (*n* = 47)	*χ* ^2^	*P*
Primary patency	6 months after operation	48 (85.71)	41 (87.23)		1.000^*∗*^
	12 months after operation	52 (92.86)	44 (93.62)		1.000^*∗*^

F-TLR	6 months after operation	51 (91.07)	36 (76.60)	4.081	0.043
	12 months after operation	44 (78.57)	28 (59.57)	4.383	0.036

Restenosis rate	6 months after operation	3 (5.36)	8 (17.02)	3.645	0.056
	12 months after operation	9 (16.07)	16 (34.04)	4.490	0.034

Limb salvage	6 months after operation	56 (100.00)	47 (100.00)	—	—
	12 months after operation	56 (100.00)	45 (95.74)		0.206^*∗*^

^*∗*^Fisher's exact probability test.

**Table 4:** Comparison of liver and kidney functions before and after surgery between the two groups (*x̅* ± *s*).

Metrics		DCB group (*n* = 56)	BMS group (*n* = 47)	*t*	*P*
ALT (U/L)	Preoperation	21.89 ± 7.64	22.25 ± 7.83	0.236	0.814
	6 months after operation	23.45 ± 6.84	23.18 ± 5.47	0.218	0.826

AST (U/L)	Preoperation	27.89 ± 8.61	27.03 ± 8.95	0.496	0.621
	6 months after operation	26.51 ± 7.74	26.63 ± 5.38	0.090	0.929

Scr (*μ*mol/L)	Preoperation	77.28 ± 14.65	76.14 ± 12.85	0.416	0.678
	6 months after operation	80.64 ± 16.49	79.21 ± 15.33	0.453	0.652

BUN (mmol/L)	Preoperation	5.76 ± 1.25	5.81 ± 1.36	0.194	0.846
	6 months after operation	5.54 ± 1.18	5.19 ± 1.82	1.175	0.243

## Data Availability

The datasets used and analyzed during the current study are available from the corresponding author upon request.
